The article "RUNX2 promotes epithelial differentiation of ADSCs and burn wound healing via targeting E-cadherin" was retracted in 2025. Reasons: manipulated images; duplicated images; unreliable data; unreliable results or conclusions.

# RUNX2 promotes epithelial differentiation of ADSCs and burn wound healing via targeting E-cadherin

**DOI:** 10.18632/oncotarget.23522

**Published:** 2017-12-21

**Authors:** Qiang Li, Han Zhao, Sizhan Xia, Hanxiao Wei, Feifei Chen, Peisheng Jin

**Affiliations:** ^1^ Department of Plastic Surgery, Affiliated Hospital of Xuzhou Medical University, Xuzhou, Jiangsu, China; ^2^ Jiangsu Center for the Collaboration and Innovation of Cancer Biotherapy, Cancer Institute, Xuzhou Medical University, Xuzhou, Jiangsu, China; ^3^ Department of Plastic Surgery, Xuzhou Central Hospital, Xuzhou, Jiangsu, China

**Keywords:** RUNX2, E-cadherin, epithelial differentiation, burn wound, ADSCs

## Abstract

Epithelial differentiation of adipose-derived stem cells (ADSCs) is mediated by sophisticated interactions of various molecular functions and biological processes, including transcriptional regulation. Runt-related transcription factor 2 (RUNX2) increases osteoblast and adipocyte differentiation of ADSCs. However, the role of RUNX2 in epithelial differentiation of ADSCs is unknown. We first showed that ADSCs possess the potential to differentiate into epithelial lineage. Then, we employed the effect of RUNX2 on epithelial differentiation of ADSCs. Our data showed that RUNX2 promoted epithelial differentiation of ADSCs. Overexpression or knockdown of RUNX2 resulted in increase or decrease of E-cadherin expression, respectively. Abatement of E-cadherin in ADSCs attenuated RUNX2-activated epithelial conversion of ADSCs and epithelial markers cytokeratin 18 (CK18) and zonula occludens protein-1 (ZO-1). We also evaluated the effect of RUNX2 on burn wound healing *in vivo*. The wound re-epithelialization were accelerated by RUNX2. The wound closure indexs, demis regeneration and revascularization were all improved. Furthermore, RUNX2 binding directly to the E-cadherin promoter region was characterized in ADSCs by chromatin immunoprecipitation (ChIP) and luciferase promoter reporter assays. Taken together, the study demonstrates the role of RUNX2 in epithelial differentiation of ADSCs and suggests that RUNX2 promotes E-cadherin expression, at least in part, through its direct binding to the promoter.

## INTRODUCTION

Burn wounds, the thermal damage to the skin, can lead to severe complications and have been demonstrated to have a devastating effect on skin functionally and cosmetically, necessitating the search for a better and more efficient cure. In recent decades, due to the introduction of treatment modalities with the application of stem cells, the regenerative medicine has been revolutionized. In the field of wound healing, the use of stem cells has been reported for curing different types of wounds [1, 2]. Moreover, studies have shown the efficacy of stem cells in promoting faster and superior burn wounds healing [3]. The use of stem cells may open up a new arena of possibilities to improve wound healing in burn patients.

Mesenchymal stem cells (MSCs) are multipotent cells capable of self-renewal and differentiation into tissue-specific cell types. Among the various sources of MSCs, ADSCs are abundant and easily obtained from subcutaneous adipose tissue via liposuction in the clinic [4, 5]. Emerging evidence has shown the beneficial effects of ADSC administration to treat various diseases because of their simple isolation techniques, easy expandability, low immunogenicity, and pluripotency [4, 6]. ADSCs possess considerable self-renewal ability and can differentiate into cells with characteristics of hepatocytes [5], neurons [7], endothelial cells [8] or renal epithelial cells [9]. In addition, ADSCs has been demonstrated to differentiate into epithelial cells to facilitate dermal wound healing [10]. The early stage of an epithelial differentiation can be observed in the existing induction system [10, 11]. Although some epithelial-specific markers have been reported to be induced in cultured ADSCs [12–14], the molecular mechanisms underlying ADSCs differentiation into the epithelial lineage are also poorly understood. Exploring the molecular mechanisms involved in ADSC differentiation is therefore of paramount importance.

More and more transcription factors are considered to involve in ADSC differentiation. RUNX2 is a member of RUNX family transcription factors, which contains a conserved motif of 128 amino acids, and is highly homologous to the Runt protein of Drosophila melanogaster [15]. The RUNX2 gene was first cloned in 1997 and is exclusively expressed in bone tissue or osteoblasts [16]. RUNX2 regulates osteogenesis directly and plays a vital role in osteoblast differentiation during embryonic development. Recently, RUNX2 is reported to play a vital role in adipocyte differentiation of mesenchymal cell [15, 17]. Furthermore, RUNX2 is shown to have great potential in regulating epithelial-mesenchymal transition (EMT), the process of which has been implicated in cancer invasiveness and metastasis [18–20]. However, the role of RUNX2 in mesenchymal-epithelial transition (MET) of ADSCs still remains unknown.

In the present study, RUNX2, E-cadherin and other epithelial differentiation markers expression were induced during early stage of epithelial differentiation. Knockdown of E-cadherin in ADSCs gave rise to downregulation of differentiation markers and epithelial differentiation. Further, RUNX2 binding site in the E-cadherin promoter directly was identified. Additionally, RUNX2 promote the therapeutic effect of ADSCs on burn wounds of nude mice. These results imply a novel role of RUNX2 in facilitating epithelial differentiation of ADSCs.

## RESULTS

### The expression of RUNX2 and E-cadherin are up-regulated during epithelial differentiation of ADSCs

In order to detect the epithelial differentiation ability of ADSCs, we first observed the cell morphology after cultured in induced medium. Phase-contrast microscopy showed a gradual conversion of ADSCs into epithelial phenotype. ADSCs without induced medium exhibited a elongated fibroblast-like morphology. After 14 days induction, cells got shorter and smaller, but still showed great difference with epithelial cells (Figure 1A).

**Figure 1:** Expression of RUNX2 and E-cadherin during epithelial differentiation **(A)** The ADSC morphology under the microscope after treatment with induced medium (×200). **(B)** Protein levels of RUNX2, E-cadherin, CK18 and ZO-1 in ADSCs during epithelial differentiation were determined by western-blot, β-actin was used as loading control. **(C)** The mRNA expression of RUNX2, E-cadherin, CK18 and ZO-1 were detected by real-time RT-PCR. Relative mRNA expressions are normalized to β-actin. **(D)** Immunofluorescence analysis to assess the expression of RUNX2, E-cadherin, CK18 and ZO-1 in ADSCs during epithelial differentiation (right panel) in comparison to control cells (left panel) (×100). Nuclei are visualized by 4,6-diamidino-2-phenylindole staining. These data are expressed as the mean ± SD (^*^P<0.05, ^**^P<0.01). Each experiment was repeated at least three times.

E-cadherin is one of the important adhesion molecules and plays a crucial role in the maintenance of epithelial integrity. We examined E-cadherin expression after induction. Data showed a faint increase of E-cadherin when ADSCs exposured to induced medium. We also assessed expression changes in other epithelial markers during the differentiation from fibroblast to epithelial cells. An initial slight increase of CK18 and ZO-1 can be observed after induction (Figure 1B–1D, Supplementary Figure 1A, 1B). Our results suggested that ADSCs possess the potential to differentiate into epithelial lineage.

### RUNX2 conducts ADSCs differentiation

RUNX2 is thought to play vital role in osteoblast and adipocyte differentiation of mesenchymal cell. In order to evaluate the role of RUNX2 in ADSCs differentiation, we first detect the expression of RUNX2 during epithelial differentiation by Western blot, qRT-PCR and immunofluorescence. Faint expression of RUNX2 was observed after the epithelial differentiation (Figure 1B–1D, Supplementary Figure 1A, 1B). Then, we added RUNX2 lentivirus into induced ADSCs for 14 days, phase-contrast microscopy displayed a gradual conversion of ADSCs into a more epithelial polygonal phenotype when RUNX2 was up-regulated (Figure 2A). Results from Western blot, qRT-PCR and immunofluorescence showed that RUNX2 was significantly up-regulated. Meanwhile, the expression of E-cadherin, CK18 and ZO-1 were also increased obviously (Figure 2C, 2E, 2G, Supplementary Figure 2A, 2B).

**Figure 2:** RUNX2 positively regulates E-cadherin expression and epithelial differentiation **(A and B)** Representative image of ADSC morphology under the microscope after ADSCs treatment with LV5-RUNX2 or LV3-shRUNX2 (×200). **(C and D)** Western blot analyses of protein levels of RUNX2, E-cadherin, CK18 and ZO-1 after ADSCs given LV5-RUNX2 or LV3-shRUNX2. β-actin was used as an internal control. **(E and F)** qRT-PCR analyses of mRNA levels of RUNX2, E-cadherin, CK18 and ZO-1 after ADSCs given LV5-RUNX2 or LV3-shRUNX2. **(G and H)** Immunofluorescence analysis to assess the expression of RUNX2, E-cadherin, CK18 and ZO-1 in ADSCs after ADSCs given LV5-RUNX2 or LV3-shRUNX2 (×100). Nuclei are stained by 4,6-diamidino-2-phenylindole. These data are expressed as the mean ± SD (^*^P<0.05, ^**^P<0.01). Each experiment was repeated at least three times.

As a complementary approach, cells were also added with RUNX2 shRNA lentivirus prior to epithelial induction. These shRNA lentivirus have been shown to efficiently knockdown RUNX2 mRNA and protein levels. Moreover, ADSCs treated with RUNX2 shRNA lentivirus showed significantly lower levels of endogenous E-cadherin (Figure 2D, 2F, 2H, Supplementary Figure 2C, 2D) and down-regulation of other epithelial marker gene was seen to be affected by RUNX2 activity. Cells still shown a flattened fibroblast-like morphology after 14 days’ induction (Figure 2B). Our results suggested a relationship between RUNX2 and E-cadherin to regulate epithelial differentiation of ADSCs.

### RUNX2 promotes ADSCs differentiation through E-cadherin

To investigate whether RUNX2 can regulate epithelial differentiation of ADSCs through E-cadherin, we first investigated the role of E-cadherin in the process of epithelial differentiation of ADSCs. E-cadherin lentivirus resulted in the high expression of E-cadherin, CK18 and ZO-1 (Figure 3C, 3E, 3G, Supplementary Figure 3A, 3B). Gradual conversion of ADSCs into epithelial polygonal phenotype could be seen in E-cadherin over-expressed group (Figure 3A). However, cells treated with E-cadherin shRNA lentivirus blocked the epithelial conversion of ADSCs. Cells still displayed a flattened fibroblast-like morphology after 14 days’ induction (Figure 3E). The expression of CK18 and ZO-1 were also inhibited by knockdown of E-cadherin expression (Figure 3D, 3F, 3H, Supplementary Figure 3C, 3D).

**Figure 3:** E-cadherin facilitate epithelial differentiation **(A and B)** Representative image of ADSC morphology under the microscope after ADSCs given LV5-E-cadherin or LV3-shE-cadherin (×200). **(C and D)** Western blot analyses of protein levels of E-cadherin, CK18 and ZO-1 after ADSCs treatment with LV5-E-cadherin or LV3-shE-cadherin. β-actin was used as an internal control. **(E and F)** qRT-PCR analyses of mRNA levels of E-cadherin, CK18 and ZO-1 after ADSCs given LV5-E-cadherin or LV3-shE-cadherin. **(G and H)** Immunofluorescence analysis of the expression of E-cadherin, CK18 and ZO-1 after ADSCs given LV5-E-cadherin or LV3-shE-cadherin (×100). Nuclei are visualized by 4,6-diamidino-2-phenylindole staining. These data are expressed as the mean ± SD (^**^P<0.01). Each experiment was repeated at least three times.

To determine whether E-cadherin is involved in RUNX2-mediated ADSCs differentiation, we suppressed E-cadherin using E-cadherin shRNA lentivirus in RUNX3-overexpressing ADSCs. E-cadherin down-regulation attenuated RUNX2-mediated epithelial conversion of ADSCs. (Figure 4A). Moreover, CK18 and ZO-1 were also abrogated by knock down of E-cadherin in RUNX3-overexpressing ADSCs (Figure 4B–4D, Supplementary Figure 4A, 4B). These results suggested that the effects of RUNX2 on ADSCs differentiation were largely dependent on E-cadherin.

**Figure 4:** RUNX2 promotes ADSCs differentiation through E-cadherin **(A)** Representative image of ADSC morphology under the microscope after ADSCs given LV5-RUNX2 or LV3-shE-cadherin (×200). **(B)** Western blot analyses of protein levels of RUNX2, E-cadherin, CK18 and ZO-1 after ADSCs given LV5-RUNX2 or LV3-shE-cadherin. β-actin was used as an internal control. **(C)** qRT-PCR analyses of mRNA levels of E-cadherin, CK18 and ZO-1 after ADSCs given LV5-RUNX2 or LV3-shE-cadherin. **(D)** Immunofluorescence analysis to assess the expression of RUNX2, E-cadherin, CK18 and ZO-1 after ADSCs given LV5-E-cadherin or LV3-shE-cadherin (×100). Nuclei are stained by 4,6-diamidino-2-phenylindole. These data are expressed as the mean ± SD (^*^P<0.05, ^**^P<0.01versus induced medium group; ^#^*P*<0.05, ^##^*P*<0.01 versus LV5-RUNX2 group). Each experiment was repeated at least three times.

### RUNX2 directly bind to the E-cadherin promoter

In order to explore the interaction of RUNX2 with E-cadherin, we analyzed the upstream region of E-cadherin and found the consensus RUNX2 binding motif (E-box sites, TCACCGCGT or CGACCGCAC) in the putative promoter (Figure 5A). To determine whether RUNX2 physically associates with this regulation region, we carried out ChIP qPCR and as shown in Figure 5B, epithelial induction significantly increased RUNX2 binding to the E-cadherin promoter region, while less binding on the promoter in Chromatin immunoprecipitation obtained with a control IgG or from cells in non-induced (-). Enrichment of RUNX2 binding was also detected in the promoter region of osteocalcin, a gene whose transcription is known to be regulated by RUNX2, and served as a positive control.

**Figure 5:** RUNX2 direct regulation on the promoter **(A)** Schematic diagram of the human E-cadherin gene promoter showing the positions of potential binding sites of putative transcription factor RUNX2 analyzed using Jarsper. Two segments at -336 bp (site1) and -579 bp (site2) upstream from the transcription start site (TSS). **(B)** Binding of RUNX2 to the E-cadherin promoter region in ADSCs cultured with epithelial differentiation medium or control (-) were detected by chromatin immunoprecipitations. Protein-chromatin crosslinked complexes were immunoprecipitated with either RUNX2 antibody or negative control antibody IgG. Chromatin immunoprecipitate obtained in the ChIP assay was quantified by real-time PCR. PCR primers spanning E-cadherin promoter including the three putative binding sites regions were employed. OCN promoter primers were used as a positive control. The data show promoter occupancy normalized to Input and represent Mean ± SD of three independent experiments, ^*^P<0.05, ^**^P<0.01. **(C)** Activity of the E-cadherin promoter in ADSCs co-transfected with the indicated amounts of pCMV-RUNX2 plasmid, pGL3- E-cadherin promoter and pRL-TK. Dose dependent increase of E-cadherin promoter activity in ADSCs with increasing concentration of pCMV-RUNX2 plasmid was measured by dual-luciferase assay. Luciferase values expressed were normalized with respect to pRL-TK value. **(D)** Induced ADSCs were transfected with pCMV vector, pCMV-RUNX2, siRNA or siRUNX2 respectively for 48 h. Total cell lysates obtained from these cells were assayed for luciferase activity and normalized with pRL-TK activity co-expressed in these cells. **(E)** Induced ADSCs were transfected with pCMV vector, pCMV-RUNX2, siRNA or siRUNX2 respectively for 48 h. Total cell lysates obtained from these cells were assayed for luciferase activity and normalized with pRL-TK activity co-expressed in ADSCs. Data represent triplicate studies with a mean ± SD. ^*^P < 0.05, ^**^P < 0.01, ^*^P < 0.05, ^***^P < 0.001. Each experiment was repeated at least three times.

To study the transcriptional activity of RUNX2 on E-cadherin promoter, transient co-transfection experiments were performed on HEK293 cells and demonstrated a dose dependent increase in E-cadherin promoter activity, with increasing concentrations of transfected pCMV-RUNX2 plasmid (Figure 5C).

To determine the potential role of RUNX2 in modulate E-cadherin gene promoter activity under epithelial stimulation, ADSCs were transiently co-transfected with pGL-E-cadherin promoter reporter plasmid with pCMV-RUNX2 or empty vector pCMV with inductive medium. We then performed a dual-luciferase transcription activation assay and our data showed that the RUNX3 binding motif (CGACCGCAC) contributed to the regulation of the E-cadherin promoter because deletion CGACCGCAC attenuated RUNX2-mediated activation (Figure 5D, 5E). Conversely, mutation of RUNX3 binding motif abrogated knockdown of RUNX2-mediated inhibition of E-cadherin promoter activity.

### RUNX2 promoted the healing of burns skin *in vivo*

To assess the effect of RUNX2 on burn wounds repairing, a 1cm in diameter degree II burn wound were created on the back of mice. ADSCs stably expressing RUNX2 or shRUNX2 were injected around wound bed. The healing area of wounds was evaluated 7 days after treatment. As shown in Figure 6A and 6B, forced expression of RUNX2 in ADSCs accelerated the wound healing of mice. The wound closure index was significantly higher in the RUNX2 high expressed group. Conversely, knock down of RUNX2 in ADSCs generated a negative effect on the burns skin. The wound closure index was the lowest when compared with other groups.

**Figure 6:** RUNX2 promotes the burn wound healing of mice **(A)** Degree II burn wound were created on the back of mice. ADSCs stably expressing RUNX2 or shRUNX2 were injected into the burn wounds. Gross appearance of the skin wounds were evaluated 7 days after treatment. **(B)** ADSCs marked with fluorescent dye CM-Dil were injected into the burn wounds, red fluorescence indicates CM-Dil-labeled ADSCs nuclei. The distribution of CM-Dil-labeled cells was observed 7 days after seeded in wound (×200). **(C)** HE staining were employed to evaluate the dermal collagen levels, fibroblast numbers and capillary density of burn wounds (×200). Data were shown as means ±SD (^*^P<0.05, ^**^P<0.01, ^***^P<0.001).

To track the differentiation of ADSCs and skin remodeling process *in vivo*, cells were prelabeled with fluorescent dye CM-Dil. The distribution of CM-Dil-labelled cells was observed 7 days after seeded in wound. We can see that few cells survived in the wound bed. No cells were observed in the dermal, subcutaneous and granulation tissue in the five groups. Most survival cells were distributed in the neo-epidermis. Moreover, cells over-expressed RUNX2 exhibited a more survival and differentiating ability. More CM-Dil-labelled cells can be found in the RUNX2 over-expressed, suggesting that RUNX2 promote ADSCs differentiation *in vivo* (Figure 6C, 6D).

HE staining of the wounds indicated that RUNX2 over-expressed ADSCs can promote skin regeneration of burn wounds, accompanying increased dermal collagen levels, fibroblast numbers and capillary density. The re-epithelization rate of ADSCs *in vivo* was significantly accelerated by RUNX2. Also, the regenerated demis of wounds were thicker at day 7. Conversely, skin regeneration of burn wounds were inhibited by knockdown of RUNX2 in ADSCs. Silencing of RUNX2 suppressed the re-epithelization rate of ADSCs *in vivo* (Figure 6E).

A immunohistochemical staining for CD31, E-cadherin and sirius red staining for collagen were also performed to evaluate the neovascularization and re-epithelialization of wound tissue. Seven days after transplantation, more CD31 positive vessel-like structures were observed in RUNX2 group but less in RUNX2 shRNA group (Figure 7A). The E-cadherin and collagen expression was also increased in RUNX2 group when compared with other four groups (Figure 7B, 7C). These data suggest that RUNX2 promote revascularization and re-epithelialization of ADSCs for burn wounds.

**Figure 7:** RUNX2 improves neovascularization and re-epithelialization of burn skin of mice **(A)** Seven days after transplantation, immunohistochemical staining for CD31 were performed to evaluate the neovascularization of wound tissue (×200). **(B)** Immunohistochemical staining for E-cadherin were performed to evaluate the effect of RUNX2 on re-epithelialization of wound tissue (×200). **(C)** Sirius red staining for collagen were employed to evaluate dermal collagen level of wound tissue (×200).

## DISCUSSION

ADSCs possess a multilineage differentiation potential and are at the forefront of cell-based therapies. Beside their well-known differentiation into cells of mesodermal origin, the potential of ADSCs’ ability to differentiate into lineages with nonmesodermal origin is even more exciting. It was reported that ADSCs can differentiate into cells with characteristics of epithelial lineage [5, 7, 11]. Nevertheless, only the early stage of an epithelial differentiation of ADSCs were discovered. CK are the first epithelial structural proteins that are expressed during epithelial differentiation [26]. ADSCs is reported to induce epidermal markers CK 5 and 14 and participate in dermal wound healing [10]. Except that, CK18 and pan CK were also be reported to be induced in ADSCs at the preliminary differentiation [9–12]. But few studies have focused on other epithelial-specific markers during epithelial differentiation of ADSCs.

In our study, we made some change on our induction system to facilitate ADSCs differentiation. Compare with induction system described by Griesche et al [22], our induction system additionally added both EGF and FGF but without bone morphogenetic protein 7 (BMP7). EGF and FGF are widely confirmed to promote ADSCs cell proliferation and epithelial differentiation [26]. However, as a member of the transforming growth factor β (TGF-β) superfamily, BMP7 negatively regulate RUNX2 expression [27]. So, we made these change to improve our induction system. As our data showed, except CK18, cell adhesion molecule E-cadherin or tight junctional protein ZO-1 were also be observed when cells were cultured in the induction medium for 14 days. These suggest that our induction system promote ADSCs differentiate towards epithelial lineage.

Cell-cell contacts are essential for the morphologic integrity of epithelial cells, as well as their control of cell proliferation and differentiation. The epithelial tissues achieve their mature organization and function partly through the formation of stable junctions between adjacent cells. Such cell-cell adhesion is controlled by adherens junctions and tight junctions [22]. As a component of adherens junctions, E-cadherin is expressed on the surface of cytoplasmatic membranes. The interaction between cytoplasmic regions of E-cadherin and catenins leads to the reorganization of actin cytoskeleton, through which diverse cell functions including cell proliferation, survival and differentiation were regulated [28]. In our study, we found that E-cadherin induced gradual conversion of ADSCs into epithelial polygonal phenotype. Knockdown of E-cadherin resulted in a flattened fibroblast-like morphology of ADSCs.

It was believed that the formation of E-cadherin junctions precede the establishment of tight junctions. As a vital component of tight junctions, ZO-1 also plays a important role in the regulation of cellular cytoskeleton, polarity and signal transduction, thus involved in the control of cell growth and differentiation [29, 30]. It has been reported that E-cadherin-catenin complexes can recruit ZO-1 to the primordial cell-cell adhesion sites. Moreover, hypoglycosylated E-cadherin is verified to result in diminished binding of ZO-1 to PP2A and increased pools of serine-phosphorylated ZO-1 [31]. Consequently, we investigated the expression of ZO-1 after up-regulation or inhibition of E-cadherin. We found that ZO-1 expression can be influenced by E-cadherin during ADSCs differentiation. Meanwhile, CK18 was also regulated coincidence with the expression of E-cadherin during epithelial differentiation regulated by E-cadherin. These results revealed that E-cadherin is involved in the epithelial differentiation of ADSCs and can regulate ZO-1 and CK18 expression.

Tissue differentiation of ADSCs is an orchestrated process requiring the physiological interplay of various factors, such as transcription factor and signaling pathway. RUNX2 is thought to be an important transcription factor which can regulate osteoblast and adipocyte differentiation of ADSCs. Runx2^−/−^ mice exhibit a complete lack of intramembranous and endochondral ossification *in vivo* and Runx2−/− calvarial cells cannot differentiate into osteoblasts, even in the presence of osteogenic factors *in vitro* [32]. Kim et al revealed that 1,25-Dihydroxyvitamin D_3_ induces the transdifferentiation of osteoblasts to adipocytes via RUNX2 downregulation in osteoblasts [33]. As an important regulator of EMT, RUNX2 showed great potential in regulating the expression of mesenchymal or epithelial markers, such as cadherin [18]. However, the role of RUNX2 in ADSCs MET is blank. In the present study, the function of RUNX2 as an epithelial differentiation regulatory factor were investigated. In fact, RUNX2 was found to be involved in the expression of E-cadherin, CK18 and ZO-1 and can promote epithelial differentiation of ADSCs. A burn wound healing assay were also conducted *in vivo* to determine the function of RUNX2. As we expected, the wound re-epithelialization were obviously accelerated by RUNX2. A re-epithelialization facilitate wound closure, demis regeneration and revascularization during the granulation tissue formation phase of wound healing. Furthermore, RUNX2 regulates E-cadherin, CK18 and ZO-1 expression. E-cadherin down-regulation by shRNA attenuated RUNX2-induced CK18 and ZO-1 up-expression and abrogated RUNX2-mediated epithelial conversion of ADSCs. These results suggested that the effects of RUNX2 on ADSCs differentiation were largely dependent on E-cadherin. were largely dependent on E-cadherin.

RUNX2 can bind the promoter of target gene to regulate its expression. Osteocalcin (OCN) is an osteoblast specific protein, regarded as a hallmark of osteoblast cells differentiation and maturation. The cis-element in the OCN gene promoter is OES2, which has an identical sequence to the Runt-binding site of RUNX2 [34]. The RUNX2 binding site was also found in the promoter of bone sialoprotein and osteopontin genes to promote osteoblast differentiation [35, 36]. We analyzed the upstream region of E-cadherin and found the consensus RUNX2 binding motif in the putative promoter. So we performed ChIP assays during epithelial differentiation and found that RUNX2 was recruited to the E-cadherin promoter with a remarkably similar temporal pattern. Dual luciferase reporter assays revealed RUNX2 increasing E-cadherin gene promoter activity in a dose dependent manner. Mutation of RUNX3 binding motif abrogated knockdown of RUNX2-mediated inhibition of E-cadherin promoter activity. These results provide evidence that RUNX2 promotes E-cadherin expression, at least in part, through its direct binding to the promoter and, possibly, other regulatory elements within the E-cadherin locus.

In conclusion, exogenous expression of RUNX2 enhanced E-cadherin expression and knockdown of RUNX2 down-regulated E-cadherin expression. RUNX2 can directly bind to the E-cadherin promoter site and activate promoter activity of E-cadherin to specifically regulate E-cadherin expression. Furthermore, RUNX2 promoted the healing of burns skin *in vivo*. These findings suggest that RUNX2 plays a critical role in improving epithelial differentiation. These results will help us to understand the role of RUNX2 in osteogenesis and may provide a new potential therapeutic target for wound skin regeneration.

## MATERIALS AND METHODS

### Isolation and culture of human ADSCs

Human ADSCs were isolated from subcutaneous adipose tissue samples obtained from the liposuction aspirates of patients undergoing cosmetic liposuction at the Affiliated Hospital of Xuzhou Medical University as previously described [21]. All of donors gave written informed consents and this study was performed using a protocol approved by the Institutional Review Board of the Affiliated Hospital of Xuzhou Medical University (Approval No. xyfylw2014030). ADSCs and HEK293 cells were maintained in DMEM containing 10% fetal bovine serum and cultured in a 37˚C humidified incubator with 95% air and 5% CO_2_. Cells from 3-6 passage were used in the following studies. Before experimental use, fluorescence-activated cell sorting analysis was conducted to detect the surface antigens CD31, CD44, CD45, CD49d, CD105 and CD106. Cells were also confirmed to possess the ability to differentiate into adipocytes and osteoblasts.

### Epithelial differentiation induction of ADSCs

The induction medium for the differentiation of ADSCs were prepared according to a previously described procedure with certain improvements [22]: L-DMEM containing 10% FBS were added with 25 μg/ml EGF, 5 μg/ml ATRA, 10 μg/ml ActA, 5 μg/ml FGF, 5 μg/ml insulin, 0.4 μg/ml hydrocortisone and 20 μg/ml glutamine. Cells were cultured in appropriate culture flasks and induction medium were transferred onto ADSCs. Cells were cultured for 14 days and medium were replaced every 3 days. The expression of epithelial markers CK18 and ZO-1 were detected by Western blot, qRT-PCR and immunofluorescence analysis.

### Transfection

The pcDNA3.1, RUNX2/pc3.1 expression plasmids were obtained from Shanghai Gene Pharma Company of China. For transient transfection of the pcDNA3.1 and RUXN2/pc3.1 plasmids into HEK293 or ADSCs were carried out using Lipofectamine 2000 transfection reagent (Invitrogen, USA) following the manufacturer's protocol. Non-specific control siRNA or RUNX3 siRNA were purchased from Integrated Biotech Solutions (Shanghai, China). The cells were transfected with siRNA using siLentFect Lipid Reagent (Bio-Rad, Hercules, CA, USA) according to the manufacturer's instructions.

For stable transfection, the lentiviral expression vectors LV5-Control, LV3-Control, LV5-RUNX2, LV5-E-cadherin, LV3-shRUNX3 and LV3-shE-cadherin were obtained from Shanghai Gene Pharma Company of China. Lentiviruses were mixed with polybrene (5 mg/ml) and added ADSCs. Positive clones were selected in puromycin (5 mg/ml). Stable transfectants were isolated after 2 weeks.

### Western blot

Cells were harvested from culture flasks. Aliquots of cell extracts were separated on a 10% SDS–polyacrylamide gel. The proteins were then transferred to nitrocellulose membrane and incubated overnight at 4˚C with following antibodies: Rabbit polyclonal anti-RUNX2 (1:1000; Cell Signaling Technology, USA), E-cadherin (1:1000), CK18 (1:1000), ZO-1 (1:1000) and β-actin (Boster, China 1:10000). Blots were washed three times with TBS containing 0.1% Tween-20 (TBST), and then incubated with horseradish peroxidase (HRP)-linked anti-rabbit secondary antibodies (1:1000; Bioworld, China) at room temperature for 2 h. After three washes with TBST, immunoreactive protein bands were detected with Tanon scanning system.

### Quantitative real-time PCR (qRT-PCR)

Total RNA extracted from cells with Trizol (Ambion, USA) was subjected to reverse transcription using the PrimeScript RT Master Mix Kit (TaKaRa, Japan). Real-time PCR analysis was performed with Power SYBR® Green PCR Master Mix (TaKaRa, Japan) for

E-cadherin: forward5′-TGGAGAGACACTGCCAACTG-3′,

reverse5′-GGCTTTGGATTCCTCTCACA-3′,

RUNX2: forward5′-GCGCATTCCTCATCCCAGTA-3′,

reverse5′- GGCTCAGGTAGGAGGGGTAA-3′,

CK18: forward5′-CAGGAATGGGAGGCATCCAG -3′,

Reverse5′-AAGTGCTCCCGGATTTTGCT-3′,

ZO-1:forward5′-AGCCATTCCCGAAGGAGTTG -3′

reverse5′-CCAACCGTCAGGAGTCATGG-3′,

β-actin: forward5′-CGGGAAATCGTGCGTGACAT-3′,

reverse5′-CGGACTCGTCATACTCCTGCTTG -3′.

### Immunofluorescence

Cells were cultured in 6-well culture dish, then fixed with 4 % paraformaldehyde and permeabilized in methanol. After washing with PBS, slides were treated with 0.2% TritonX-100 in PBS and incubated with primary antibody (Cell Signaling Technology, USA, RUNX2, 1:50; E-cadherin, 1:50, CK-18, 1:50, ZO-1, 1:50) overnight at 4°C. Then cells were incubated with secondary antibody (Alexa flour 594-conjugated goat anti-mouse IgG, flour 594-conjugated goat anti-rabbit IgG, Thermo Fisher scientific, USA) for 2 hours at 37˚C (1:100). The slides were mounted with 4,6-diamidino-2-phenylindole and analyzed by a Nikon fluorescence microscopeand images were captured by Nikon camera.

### Chromatin immunoprecipitation

Cells transfected with control or RUNX2 plasmids were cross-linked by incubation in 1% (v/v) formaldehyde-containing medium for 10 min at 37°C, then sonicated to form soluble chromatin. A RUNX2 antibody was used to precipitate DNA fragments bound by their corresponding elements. The protein-DNA complex was collected using protein A Agarose (Millipore, USA) and then eluted and reverse cross-linked. After protease K treatment, samples were extracted with phenol/chloroform and precipitated with ethanol. Recovered DNA was re-suspended in TE buffer and amplified by PCR. Primers used for ChIP assay were as follows:

Forward: 5′-CCAGGTCTTAGTGAGCCACC-3′

Reverse: 5′-CGTACCGCTGATTGGCTGAG-3′.

### Reporter vector construction and luciferase reporter assay

To generate the pGL3-E-cadherin promoter construct, the fragment of E-cadherin promoter was PCR amplified from mouse genomic DNA using High Fidelity polymerase (Takara, Japan). The fragment was cloned directionally between Hind III and Xho I sites of pGL3 basic vector (Promega). The RUNX2 binding sequence at the human E-cadherin gene and putative E-cadherin promoter was created by PCR and subsequent cloned into pGL3 vector.

HEK293T cells were co-transfected with pCMV-RUNX2 plasmid of gradual increase dose from 100 ng to 400 ng and pGL3-E-cadherin promoter constructs. ADSCs were transiently transfected with appropriate reporter plasmids and RUNX2, control plasmids, siRNA for RUNX2 or control siRNA. Cells were harvested and lysed after 48 h. Luciferase activity was measured using the Dual-Luciferase Reporter Assay System (Promega, Madison, WI, USA), normalized to renilla luciferase.

### Dermal burn model

The dermal burn models were established according to a previously described procedure with certain improvements [23, 24]. All animal studies were approved by Animal Care and Use Committee. Nude mice used in the experiment were fed in specific pathogen free individual ventilated cages. No animal was severely ill or died prior to the experimental endpoint. After anesthetizing, animals with intraperitoneal injections of chloral hydrate (10%, 5ml/Kg), a 1cm in diameter columniform iron was immersed into burning water for 1min, the degree III burn wound were created on the back of mice by putting the top of the iron on the skin for 20s.

Cells stably transfected with RUNX2 or RUNX2 shRNA were prelabeled with fluorescent dye CM-Dil (Invitrogen, USA) at 37°C for 20 min before seeded in wound. The labelled cells were rinsed and resuspended in PBS and 14×10^6^ ADSCs were injected around wound bed. The animals were sacrificed 7 days after treatment and wounds were harvested with the surrounding tissue.

### Wound repair analysis

The wound area was analyzed 7 days after treatment by tracing wound margin and calculating the area using Image J software (version 1.38; National Institutes of Health, Bethesda, MD, USA). Wound closure rate was measured as follows: Wound closure index (%) = (original wound area - unhealed wound area)/original wound area) ×100%. Tissue specimens were fixed and sections were stained with HE for light microscopy.

### Immunohistochemistry

The immunohistochemistry staining was performed as previously described [25]. The 4 μm sections were incubated with E-cadherin (1:50), CD31 (1:50) and collagen (1:50) antibody (Cell Signaling Technology, USA) and diaminobenzidine was used to produce a brown precipitate. Images were collected by a Camedia Master C-3040 digital camera.

### Sirius red staining

The slides were incubated with a 0.1% Sirius Red solution dissolved in acqueous saturated picric acid for 1 hour, washed in acidified water (0.5% hydrogen chloride). After washing with PBS, slides were treated with hematoxylin staining solution for 10 min. The slides were observed using light microscopy (Olympus BX-51 light microscope).

### Statistical analysis

Data are expressed as the mean ± SD. Two-factor analysis of variance and the Dunnett's t-test were used to assess differences within treatment groups. Values of *P*< 0.05 were considered statistically significant.

## SUPPLEMENTARY MATERIALS FIGURES



## Abbreviations

ADSCs: Adipose-derived stem cells
MSCs: Mesenchymal stem cells
RUNX2: Runt-related transcription factor 2
CK18: Cytokeratin 18
ZO-1: Zonula occludens protein-1
ChIP: Chromatin immunoprecipitation
EMT: Epithelial-mesenchymal transition
MET: Mesenchymal-epithelial transition
qRT-PCR: quantitative real-time PCR
3′UTR: 3′untranslated region.
